# Anticancer and Cytotoxicity Activity of Native and Modified Black Rice Flour on Colon Cancer Cell Lines

This article has been retracted.

**DOI:** 10.1155/2022/8575026

**Published:** 2022-02-21

**Authors:** B. Thanuja, R. Parimalavalli, S. Vijayanand, Reem Mohammed Alharbi, Neveen Abdel-Raouf, Ibraheem Borie M. Ibraheem, Essam Nageh Sholkamy, Kaliannan Durairaj, Kibrom Meansbo Hadish

**Affiliations:** ^1^Department of Food Science and Nutrition, Periyar University, Salem 636 011, Tamil Nadu, India; ^2^Department of Biotechnology, Thiruvalluvar University, Serkadu, Vellore, India; ^3^Department of Biology, College of Science, University of Hafer Al-Baten, Hafer Al-Baten, Saudi Arabia; ^4^Department of Biology, College of Science and Humanities, Prince Sattam Bin Abdulaziz University, Al-Kharj 11942, Saudi Arabia; ^5^Department of Botany and Microbiology, Faculty of Science, Beni-Suef University, Beni-Suef 65211, Egypt; ^6^Department of Botany and Microbiology, College of Science, King Saud University, Riyadh 11451, Saudi Arabia; ^7^Zoonosis Research Center, School of Medicine, Wonkwang University, Iksan, Republic of Korea; ^8^Faculty of Mechanical Engineering, AMIT Campus, Arba Minch University, Arba Minch, Ethiopia

## Abstract

This study is intended to evaluate the cytotoxicity of native and dual-modified black rice flour against the colon cancer cell line (HCT116) and mouse embryo cell line (3T3-L1) by using the MTT assay. The modification techniques applied to prepare rice flour samples were enzymatic modification and heat moisture treatment. In this study, the IC50 of native black rice flour and modified black rice flour was 255.78 *µ*g/mL and 340.85 *µ*g/mL, respectively. The result confirms that the native black rice flour has significant cytotoxic and anticancer potential against human colon cancer cells. In addition, the IC50 of native black rice flour and modified black rice flour on the 3T3-L1 cell line was found to be 345.96 *µ*g/mL and 1106.94 *µ*g/mL, respectively. The results showed that the native black rice flour had weak cytotoxicity, and modified black rice flour was nontoxic in both the cell lines. The active component of phytochemicals present in black rice flour has a potential role in preventing colon cancer.

## 1. Introduction

Worldwide, cancer is one of the health concerns. One in eight deaths worldwide is due to cancer [1]. There is a prime need to reduce the threat of this disease, especially in developing countries where the prevalence and incidence of this disease are expected to increase in the future. When we consider the risk factors, genetic defects account for only 5–10% of most cancers. In contrast, more than 90% are due to modifiable risk factors such as environmental and lifestyle factors [2, 3]. Several earlier findings proved that most human cancers could be prevented through appropriate lifestyle and dietary approaches [4]. The term “carcinogenesis” is a multistage process comprising phases such as initiation, promotion, and progression. The vital goal of chemoprevention is to block tumor progression [5].

An imbalance between pro-oxidants and antioxidants causes oxidative stress and leads to the constant and unregulated generation of reactive oxygen species, which are involved in the phases of carcinogenesis [6, 7]. Diet is recognized as a significant modulator in the development of colon cancer; high consumption of plant foods such as vegetables, fruits, and whole grains containing bioactive phytochemicals has been linked to a decreased risk of colon cancer [8]. As a result, identifying plant food sources and their bioactive components that target oxidative stress is an essential parameter for colon cancer prevention and treatment strategies. Especially among cereal grain varieties, rice is consumed as a staple food by around fifty percent of the world's population and a significant portion of the Indian population. When contrasted to polished white rice, colored rice variants are valued due to their health advantages. Compared with white rice, colored rice varieties with bran are more nutritious [9]. It has been shown that pigmented rice types have large quantities of antioxidant chemicals and have good antioxidant capabilities [10]. Due to high levels of dietary fiber, flavonoids, phenolic compounds, and anthocyanins, pigmented rice varieties such as black rice are considered and proven to be high in functional activities and produce health-promoting benefits in the human body [11].

Black rice is also high in dietary fiber and has been proven to have a decreased cancer risk. Especially black rice is linked to a reduced risk of colon cancer due to its high fiber composition, as fiber attaches to carcinogenic compounds and helps eliminate them from the body [12]. In vivo and epidemiological studies indicate that anthocyanins, which are rich in black rice, exhibit an anticarcinogenic effect [13]. Previous studies have reported that black rice has a higher anthocyanin content (428.38 mg/100 g) than other rice varieties [14].

Chemopreventive drugs could inhibit the growth of cancer cells, but it was proved in many studies that it had the side effects of drug therapy. Hence, the dietary approach plays a vital role in preventing and managing many types of cancer. Being an antioxidant-rich source, black rice displays encouraging results in cancer prevention [15]. This study was carried out to evaluate the cytotoxicity of native and modified black rice flour on normal cells (3T3-L1) and to know the anticancer effects of native and modified black rice flour on colon cancer cell lines (HCT116).

## 2. Materials and Methods

### 2.1. Raw Materials and Sample Preparation

Raw black rice was procured from the local organic market in Tiruchirappalli district, Tamil Nadu, India. Obtained rice was ground separately in the analytical mill and passed through a 100 mesh (150 *µ*m) sieve. The prepared rice flour was stored in an airtight container at 4°C for subsequent experiments. This sample was termed native black rice flour. The native rice flour was wet-milled to produce 10% moisture content and adjusted to pH 4.5 with a buffer of 0.1 M sodium acetate for preparing modified black rice flour. Then, the alpha-amylase enzyme (0.2 g) was added to the flour. Flour was incubated in a shaking water bath at 55°C for 24 hours [15] and then centrifuged (3000 g) for 10 min. Following this, the precipitate was collected by centrifugation by washing twice with distilled water. Then, it was oven-dried at 40°C for 25% of its moisture content. The samples were sealed in a container to store at room temperature for 24 hrs. Then, for about one hour, the containers were placed in a hot air oven at 100°C. The flour was sieved to obtain a 100 mesh (150 *µ*m) particle size and stored at 4°C. The modification methods applied were enzymatic modification and heat moisture treatment.

### 2.2. Extraction of Sample

One gram of each sample variety was dissolved in 25 mL of methanol solvent and kept in a shaking incubator for 24 h [16]. The extracts were filtered using No.1 Whatman filter paper and stored at a temperature of 4°C until analysis.

### 2.3. Cell Lines and Culture Medium

A human colorectal adenocarcinoma cell line (HCT116) and mouse embryo fibroblast cell line (3T3-L1) were obtained from the National Centre for Cell Science (NCCS), Pune, Maharashtra, India [17]. Maintenance of cells was carried out in a CO_2_ incubator at a pH of 7, at a temperature of 37 ± 0.5°C, and with a relative humidity of 80% as an appropriate environment for the maintenance of cells. The culture medium DMEM high glucose (#AL111, HiMedia) was also incubated for about 24–72 h.

### 2.4. MTT Assay

The MTT assay is a colorimetric method that involves measuring the reduction of yellow 3-(4, 5-dimethylthiazol-2-yl)-2, 5-diphenyl tetrazolium bromide (MTT) by mitochondrial succinate dehydrogenase. The principle is based on the number of cells present and the assumption that those dead cells or their products do not reduce tetrazolium. The MTT enters into the mitochondria in the cells and is reduced to purple-colored formazan crystals, which are insoluble. The cells were solubilized with dimethyl sulfoxide (DMSO) and then released; the solubilized formazan reagent was measured spectrophotometrically at 570 nm. Cell viability was evaluated by the MTT assay with a human colorectal adenocarcinoma cell line (HCT116) and a mouse embryo fibroblast cell line (3T3-L1) with native and modified black rice flour (25, 50, 100, 200, and 400 *µ*g/mL) compared with cell control and standard control. Cells were counted by haemocytometer and seeded at a density of 5.0 × 103 cells/well in 100 *μ*L of media in a 96-well plate culture medium and incubated overnight at 37°C. After incubation, take off the old media and add new media containing 100 *µ*L with different concentrations of the test compound in representative wells in 96 plates. The optical density of solubilized crystals in DMSO was measured at 570 nm on a microplate reader. Using the following formula, the percentage growth inhibition was calculated. The test drug concentration required to inhibit cell growth by 50% is obtained with origin software from the dose-response curves for each cell line.

(1) $$\begin{array}{c} \text{Percentage of cell viability}=\frac{\text{mean absorbance of sample}-\text{blank}}{\text{mean absorbance of untreated}-\text{blank}}\times 100. \end{array}$$

The 50% inhibitory concentrations (IC50) were calculated from five concentrations of the extracts (25, 50, 100, 200, and 400 *μ*g/mL). By applying the linear regression equation, the IC50 value was determined, i.e., *Y* = *Mx* + *C* [18]. Here, *Y* = 50, *M* and *C* values were derived from the viability graph.

### 2.5. Cell Morphology Observation

The effects of rice extracts on the cellular morphological changes were determined using the standard procedures. In this method, the effective dosage concentration of the extract is based on the inhibition concentration (IC50) value determined using the MTT assay. The morphological observation was performed at 37°C for 24 h (25, 50, 100, 200, and 400 *µ*g/mL) using a light inverted microscope (Nikon, Japan) at a magnification of 40X.

## 3. Results and Discussion

### 3.1. Cytotoxicity Assay against HCT116 Cell Lines

The 3-(4, 5-dimethylthiazol-2-yl)-2, 5-diphenyltetrazolium bromide (MTT) assay is a technical and simple method that measures the viability of cells used to screen antiproliferative agents (15). Different doses of NBRF and DMBRF extracts (methanol), ranging from 25–400 *μ*g/mL, were applied against the human colorectal adenocarcinoma cell line (HCT116). The results showed that the extracts had cytotoxicity activity on colon cancer cell lines.  Figure 1 shows in vitro cell viability assay of native and modified black rice flour against HCT-116 cell lines for 24 h.

The concentration of NBRF and DMBRF were increased, but the cell viability was decreased, ranging from 96.69 to 32.72%. The findings of the study indicate that when the concentration of black rice increased, the viability of cancer cells decreased. Overall, in all the concentrations, the native black rice flour had the highest anticancer activity when compared to modified black rice flour. Due to enzymatic and healing moisture treatment, it resulted in the loss of phytochemicals and antioxidants in modified black rice flour. A previous study reported that dual-modified black waxy and red jasmine rice flour resulted in decreased antioxidants when compared with native varieties [17].

The anticancer activity of the native and modified black rice flour is indicated as IC50, which is the concentration causing 50% of cellular proliferation inhibition. In this study, the IC50 of native and modified black rice flour was 255.78 *µ*g/mL and 340.85 *µ*g/mL, respectively (Figure 2). The result confirms that the native black rice flour has significant cytotoxic and anticancer potential against human colon cancer cells.

Originally, the phase-contrast microscopic observation displayed the morphological changes in the native and modified black rice flour-treated cancer cells. The morphological characteristic alterations in apoptotic cells were commonly applied for apoptosis detection and quantification [19]. Thus, the inverted phase-contrast microscope was used to visualize the morphological alterations that identify apoptosis. In this study, in contrast to control cells, cytomorphological changes in HCT-116 cells were identified after 24 h of treatment with tested native and modified black rice flour. The untreated cells maintained their original morphology, which included many nucleoli. The majority of the control cells remained attached to the Petri dishes of tissue culture.  Figure 3 presents cytomorphological analysis on phase-contrast microscopic images of HCT116. Similarly, Figure 4 shows cytomorphological analysis of phase-contrast microscopic images of HCT116.

The most noticeable morphological changes after revealing cells to 200 *μ*g/mL and 400 *μ*g/mL treated concentrations of native and modified black rice flour counting cells were contraction, cytoplasmic compression, and nuclear chromatin condensation. Cells enduring apoptosis resulted in different sorts of morphology and its alterations, such as echinoid spikes on the surface of apoptotic cells, apoptotic bodies, and cell number decreases, when the dosage of the native and modified black rice flour was raised. The apoptotic cells lost cellular adherence to the substrate, and the majority of the cells separated from the surface of the tissue culture dish plate and floated in the culture medium.

### 3.2. Cytotoxicity Assay against 3T3-L1 Cell Lines

The cell viability of native black rice and modified black rice was evaluated using MTT assay on a mouse embryo fibroblast cell line (3T3-L1) cell line.  Figure 5 shows a graph of the percentage cell viability on 3T3-L1 cells against different concentrations (25–400 *µ*g/mL) of the prepared systems. MTT results confirmed that the native and modified black rice flour showed no toxic effect on 3T3-L1 (mouse embryo fibroblast) cells. Even in the highest concentrations, 200 and 400 *µ*g/mL, the cell viability was recorded as 62% and 47%, respectively. In the case of modified black rice flour, in the highest concentrations, 200 and 400 *µ*g/mL cell viability were recorded as 88% and 82%, respectively. The modified black rice flour had high cell viability when compared to native black rice flour.  Figure 5 shows in vitro cell viability assay of native and modified black rice flour against 3T3-L1 cell lines for 24 h.

As per the National Cancer Institute (NCI) and the GERAN Protocol, strong cytotoxic effects are defined as IC50 values of <21 *μ*g/ml, moderate cytotoxic effects as IC50 values of 21–200 *μ*g/ml, and weak cytotoxic effects as IC50 values of 201–500 *μ*g/ml. If IC50 values are greater than 501 *μ*g/ml, they are considered noncytotoxic [20]. In our study, the IC50 value of native and modified black rice flour against the 3T3-L1 cell line was found to be 345.96 *µ*g/mL and 1106.94 *µ*g/mL, respectively (Figure 6). Therefore, according to the NCI, native black rice flour has weak cytotoxicity, and modified black rice flour is nontoxic [18, 21].

The phase-contrast microscopic display showed the different concentrations of native and modified black rice flour treated normal cells. The results revealed that there were no morphological changes that occurred in treated and untreated 3T3-L1 cells [22].  Figure 7 shows cytomorphological analysis by phase-contrast microscopic images of 3T3-L1. Similarly, Figure 8 shows cytomorphological analysis of phase-contrast microscopic images of 3T3-L1.

Black rice is rich in anthocyanins. Anthocyanins are unstable molecules because their stability is influenced by factors such as heat, chemical structure, concentration, pH, light, oxygen, solvents, enzymes, metallic ions, flavonoids, and proteins [23]. Temperature and heating duration had a strong correlation with total anthocyanin concentration and total antioxidant activity [24]. When exposed to heat or temperature, anthocyanins tend to degrade into smaller forms that are stable and could or could not have antioxidant potential [21, 25]. The findings of the result proved the impact of modification techniques (enzymatic and heat moisture treatment) applied on native black rice flour. However, this novel approach has its application in food processing and food product development.

## 4. Conclusion

Both native and modified black rice flour exhibited cytotoxicity and proved to be beneficial as anticancer agents. The findings of the result proved the impact of modification techniques (enzymatic and heat moisture treatment) applied on native black rice flour. However, this novel approach has its application in food processing and food product development. The observations strongly suggest that when compared with modified black rice flour, native black rice flour may have possible therapeutic potential against human colon cancer cells. This is supported by the results of cytomorphological changes in HCT-116 cells that were identified after 24 h of treatment with tested native and modified black rice flour. This may be due to the effects of methods applied on antioxidant content and properties. These findings provide important information to improve health and prevent cancer by improving the consumption of black rice and its products and its application in food product development.

## Figures and Tables

**Figure 1:** In vitro cell viability assay of native and modified black rice flour against HCT116 cell lines for 24 h.

**Figure 2:** IC50 values of native and modified black rice flour against HCT116.

**Figure 3:** Cytomorphological analysis on phase-contrast microscopic images of HCT116. (a) Control; (b) native black rice flour treated with 25 *μ*g/mL; (c) native black rice flour treated with 50 *μ*g/mL; (d) native black rice flour treated with 100 *μ*g/mL; (e) native black rice flour treated with 200 *μ*g/mL; and (f) native black rice flour treated with 400 *μ*g/mL.

**Figure 4:** Cytomorphological analysis of phase-contrast microscopic images of HCT116. (a) Control; (b) modified black rice flour treated with 25 *μ*g/mL; (c) modified black rice flour treated with 50 *μ*g/mL; (d) modified black rice flour treated with 100 *μ*g/mL; (e) modified black rice flour treated with 200 *μ*g/mL; and (f) modified black rice flour treated with 400 *μ*g/mL.

**Figure 5:** In vitro cell viability assay of native and modified black rice flour against extracts on 3T3-L1 cell lines for 24 h.

**Figure 6:** IC50 values of native and modified black rice flour against 3T3-L1.

**Figure 7:** Cytomorphological analysis by phase-contrast microscopic images of 3T3-L1. (a) Control; (b) native black rice flour treated with 25 *μ*g/mL; (c) native black rice flour treated with 50 *μ*g/mL; (d) native black rice flour treated with 100 *μ*g/mL; (e) native black rice flour treated with 200 *μ*g/mL; and (f) native black rice flour treated with 400 *μ*g/mL.

**Figure 8:** Cytomorphological analysis of phase-contrast microscopic images of 3T3-L1. (a) Control; (b) modified black rice flour treated with 25 *μ*g/mL; (c) modified black rice flour treated with 50 *μ*g/mL; (d) modified black rice flour treated with 100 *μ*g/mL; (e) modified black rice flour treated with 200 *μ*g/mL; and (f) modified black rice flour treated with 400 *μ*g/mL.

## Data Availability

The data used to support the findings of this study are included in the article. Should further data or information be required, request should be made to the corresponding author.

## References

[1] vel Szic K. S., Palagani A., Hassannia B. (2011). Phytochemicals and cancer chemoprevention: epigenetic friends or foe?. *Phytochemicals—Bioactivities and Impact on Health*.

[2] Tantamango-Bartley Y., Jaceldo-Siegl K., Fan J., Fraser G. (2013). Vegetarian diets and the incidence of cancer in a low-risk population. *Cancer Epidemiology Biomarkers & Prevention*.

[3] Willett W. C. (2002). Balancing life-style and genomics research for disease prevention. *Science*.

[4] Lin W.-L., Liang W.-H., Lee Y.-J., Chuang S.-K., Tseng T.-H. (2010). Antitumor progression potential of caffeic acid phenethyl ester involving p75NTR in C6 glioma cells. *Chemico-Biological Interactions*.

[5] Valko M., Leibfritz D., Moncol J., Cronin M. T. D., Mazur M., Telser J. (2007). Free radicals and antioxidants in normal physiological functions and human disease. *The International Journal of Biochemistry & Cell Biology*.

[6] Klaunig J. E., Wang Z. (2018). Oxidative stress in carcinogenesis. *Current Opinion in Toxicology*.

[7] Fernández-Villa T., Álvarez-Álvarez L., Rubín-García M., Obón-Santacana M., Moreno V. (2020). The role of dietary patterns in colorectal cancer: a 2019 update. *Expert Review of Gastroenterology & Hepatology*.

[8] Zhang L., Hu P., Tang S., Zhao H., Wu D. (2005). Comparative studies on major nutritional components of rice with a giant embryo and a normal embryo. *Journal of Food Biochemistry*.

[9] Laokuldilok T., Shoemaker C. F., Jongkaewwattana S., Tulyathan V. (2011). Antioxidants and antioxidant activity of several pigmented rice brans. *Journal of Agricultural and Food Chemistry*.

[10] Min B., McClung A. M., Chen M.-H. (2011). Phytochemicals and antioxidant capacities in rice brans of different color. *Journal of Food Science*.

[11] Deng G.-F., Xu X.-R., Zhang Y., Li D., Gan R.-Y., Li H.-B. (2013). Phenolic compounds and bioactivities of pigmented rice. *Critical Reviews in Food Science and Nutrition*.

[12] Steinmetz K. A., Potter J. D. (1991). Vegetables, fruit, and cancer. I. epidemiology. *Cancer Causes & Control*.

[13] Kristamtini T., Basunanda P., Murti R. H. (2014). Genetic variability of rice pericarp color parameters and total anthocyanine content of eleven local black rice and their correlation. *Ilmu Pertanian*.

[14] Yeh A.-I. (2004). Chapter 17: preparation and applications of rice flour. *In Book: RICE: Chemistry and Technology*.

[15] Tananuwong K., Tewaruth W. (2010). Extraction and application of antioxidants from black glutinous rice. *Lebensmittel-Wissenschaft und -Technologie- Food Science and Technology*.

[16] Franchi G. C., Moraes C. S., Toreti V. C., Daugsch A., Nowill A. E., Park Y. K. (2012). Comparison of effects of the ethanolic extracts of brazilian propolis on human leukemic cells as assessed with the MTT assay. *Evidence-Based Complementary and Alternative Medicine*.

[17] Mazewski C., Liang K., Gonzalez de Mejia E. (2018). Comparison of the effect of chemical composition of anthocyanin-rich plant extracts on colon cancer cell proliferation and their potential mechanism of action using in vitro, in silico, and biochemical assays. *Food Chemistry*.

[18] Chang H., Mi M., Ling W. (2008). Structurally related cytotoxic effects of flavonoids on human cancer cells in vitro. *Archives of Pharmacal Research*.

[19] Moongkarndi P., Kosem N., Kaslungka S., Luanratana O., Pongpan N., Neungton N. (2004). Antiproliferation, antioxidation and induction of apoptosis by garcinia mangostana (mangosteen) on SKBR3 human breast cancer cell line. *Journal of Ethnopharmacology*.

[20] Thuret G., Chiquet C., Herrag S. (2003). Mechanisms of staurosporine induced apoptosis in a human corneal endothelial cell line. *British Journal of Ophthalmology*.

[21] Brady H. J. (2004). *Apoptosis Methods and Protocols*.

[22] Saikia S., Dutta H., Saikia D., Mahanta C. L. (2012). Quality characterisation and estimation of phytochemicals content and antioxidant capacity of aromatic pigmented and non-pigmented rice varieties. *Food Research International*.

[23] Cavalcanti R. N., Santos D. T., Meireles M. A. A. (2011). Non-thermal stabilization mechanisms of anthocyanins in model and food systems—an overview. *Food Research International*.

[24] Patras A., Brunton N. P., Da Pieve S., Butler F. (2009). Impact of high pressure processing on total antioxidant activity, phenolic, ascorbic acid, anthocyanin content and colour of strawberry and blackberry purées. *Innovative Food Science & Emerging Technologies*.

[25] Yue X., Xu Z. (2008). Changes of anthocyanins, anthocyanidins, and antioxidant activity in bilberry extract during dry heating. *Journal of Food Science*.

